The article "Sensor Technology and Intelligent Systems in Anorexia Nervosa: Providing Smarter Healthcare Delivery Systems" was published in 2022. Journal: Biomed Res Int.

# Sensor Technology and Intelligent Systems in Anorexia Nervosa: Providing Smarter Healthcare Delivery Systems

**DOI:** 10.1155/2022/1955056

**Published:** 2022-09-19

**Authors:** Carlos A. Almenara, Silvia Cimino, Luca Cerniglia

**Affiliations:** ^1^School of Health Sciences, Universidad Peruana de Ciencias Aplicadas, Avenida Alameda San Marcos 11, Chorrillos, 15067, Lima, Peru; ^2^Department of Dynamic and Clinical Psychology and Health Studies. Sapienza, University of Rome Via degli Apuli, 1, 00186 Rome, Italy; ^3^Faculty of Psychology, International Telematic University Uninettuno, Corso Vittorio Emanuele II, 39, 00186 Rome, Italy

## Abstract

Ubiquitous technology, big data, more efficient electronic health records, and predictive analytics are now at the core of smart healthcare systems supported by artificial intelligence. In the present narrative review, we focus on sensing technologies for the healthcare of Anorexia Nervosa (AN). We employed a framework inspired by the Interpersonal Neurobiology Theory (IPNB), which posits that human experience is characterized by a flow of energy and information both within us (within our whole body), and between us (in the connections we have with others and with nature). In line with this framework, we focused on sensors designed to evaluate bodily processes (body sensors such as implantable sensors, epidermal sensors, and wearable and portable sensors), human social interaction (sociometric sensors), and the physical environment (indoor and outdoor ambient sensors). There is a myriad of man-made sensors as well as nature-based sensors such as plants that can be used to design and deploy intelligent systems for human monitoring and healthcare. In conclusion, sensing technologies and intelligent systems can be employed for smarter healthcare of AN and help to relieve the burden of health professionals. However, there are technical, ethical, and environmental sustainability issues that must be considered prior to implementing these systems. A joint collaboration of professionals and other members of the society involved in the healthcare of individuals with AN can help in the development of these systems. The evolution of cyberphysical systems should also be considered in these collaborations.

## 1. Introduction

Ubiquitous technology, big data, more efficient electronic health records, and predictive analytics are now at the core of smart healthcare systems supported by artificial intelligence (AI) [1]. Particularly, the advances in health informatics and sensor technology provide several possibilities for a positive transformation of traditional medical treatments. For example, intelligent systems can provide real-time feedback to electronic devices, the patient, and the physician to improve the efficiency in healthcare, reduce costs, relieve the burden of health professionals, and more importantly, to enhance human decision making, allowing better and more informed medical decisions for an optimal treatment [2]. In the present narrative review, we focus on sensing technologies for the healthcare of Anorexia Nervosa (AN). Although AN is among the least common mental disorders, AN affects approximately 13.6 million people [95% UI: 10.2–17.5 million], mostly women, and accounts for the most deaths among eating disorders [3–5]. Moreover, the illness course in AN is usually a protracted course that can develop into a severe-enduring condition with detrimental effects in the health of millions of women [6, 7].

The article "Sensor Technology and Intelligent Systems in Anorexia Nervosa: Providing Smarter Healthcare Delivery Systems" was published in 2022. Journal: Biomed Res Int.

Instead of a deep dive into the technical aspects of sensor technology, which is not our area of competence, we provide an overview of sensing technologies for researchers and health professionals in the field of eating disorders. Those interested to further explore this technology can use the extensive list of bibliographic references used to elaborate this manuscript.

This study is divided into two major sections. In the first section, we introduce sensor technology and the framework we will use to group the large diversity of sensors. This first section covers body sensors (implantable, epidermal, wearable, and portable), sociometric sensors, and ambient sensors. The second section is dedicated to the implementation of intelligent systems for smarter healthcare.

### 1.1. Sensor Technology

In general terms, sensors capture and quantify physical phenomena such as temperature [8, 9]. There is a myriad of sensors for various fields such as aerospace technology, agriculture, food packaging, and healthcare, among many others. For example, conventional electrochemical biosensors can detect biofluids in the human body like lactate [10]. More advanced biosensors, based on quantum mechanics and nanomaterials (e.g., polymer, graphene, carbon), can detect neurotransmitters like dopamine or serotonin [11–17]. For example, quantum sensors can be used to detect photons or electromagnetic fields at the atomic level, allowing the detection of neural activity [9].

Therefore, to explore the applications of sensors for the healthcare of AN, we employed a framework inspired by Interpersonal Neurobiology Theory (IPNB) [18]. IPNB posits that human experience is characterized by a flow of energy and information both within us (within our whole body), and between us (in the connections we have with others and with nature) [18]. In this regard, what we call mind, would be “the emergent, self-organizing, embodied, and relational process that regulates the flow of energy and information” ^[18(p. 4)]^. In line with this framework, we focus on sensors designed to evaluate bodily processes (body sensors), human social interaction (sociometrics), and the physical environment.

The article "Sensor Technology and Intelligent Systems in Anorexia Nervosa: Providing Smarter Healthcare Delivery Systems" was published in 2022. Journal: Biomed Res Int.

#### 1.1.1. Body Sensors

Body sensors can be further divided into different categories. In this review, we categorize them as implantable (injectable, insertable, or ingestible), epidermal (skin-attached), and wearable and portable [19].

*(1) Implantable Sensors*. The cardiac pacemaker developed in the 1960s is an illustrative example of one of the first implantable sensors [19]. Novel heart monitoring devices include Mobile Cardiac Outpatient Telemetry (MCOT; CardioNet, Inc.), Reveal LINQ (Medtronic), and Implantable Cardioverter Defibrillators (ICDs) such as Visia AF devices (Medtronic) for the management of tachyarrhythmia. Cardiovascular issues in AN are widely recognized and “are the main cause of morbidity and mortality in AN” [20]. Studies report elevated heart rate variability (HRV), bradycardia, and QT interval prolongation (that is, from the Q wave to the end of the T wave in an electrocardiogram), the latter two associated with the development of ventricular arrhythmias [20, 21].

In this regard, a recent study reported a sensor capable of providing interoceptive stimulation to enhance HRV [22]. Interoception deficits (i.e., the difficulty to accurately identify internal physiological signals like hunger or satiety), have been identified as a key symptom in network analysis of AN psychopathology [23]. Therefore, there is a venue for further research on the autonomic nervous system in AN [24] using sensing technology.

Implantable sensors can also be used for neural sensing (e.g., brain neural recording), intracranial neurostimulation (invasive deep brain stimulation, DBS), neuromodulation, and neurofeedback [25–36]. The neuroanatomical areas of major interest for the treatment of AN have been the brain's subcallosal cingulate cortex and the nucleus accumbens [36–40]. Other reports include the dorsolateral prefrontal cortex (DLPFC) [26], the bed nucleus of the stria terminalis [41], and the ventral anterior limb of the capsula interna [42]. Most of these studies have focused on eating behavior and weight gain as indicators of successful outcomes [43], and much less on body image issues ^[e.g., 40]^. First, it is important to recognize that weight gain is just one of many other important markers of a successful treatment outcome [33]. Second, it is also worth noting the caveats of implementing intracranial sensors (e.g., undergoing neurosurgery, using durable and flexible biocompatible materials, cytotoxicity) [34], and most importantly the ethical concerns that can generate these interventions [44, 45].

The article "Sensor Technology and Intelligent Systems in Anorexia Nervosa: Providing Smarter Healthcare Delivery Systems" was published in 2022. Journal: Biomed Res Int.

Implantable brain sensing technologies have raised many interests among scholars, health professionals, patients, business companies, and the public through the media depiction of brain-computer interfaces [46]. However, it has raised concerns about ethical issues related to the use and misuse of neurotechnologies [44, 47–55]. In this regard, it is important to consider both ethical issues and future directions, prior to adopting implantable neural devices and neurostimulation [56–58].

Other than heart and brain sensors, there are also implantable biosensors for tracking diverse biochemical substances and processes in the human body. There are several chemical substances of interest (biomarkers) for the treatment of AN. For example, individuals with AN commonly present an endocrine dysregulation associated with the hypothalamic-pituitary axis, and more precisely the hypothalamic-pituitary-gonadal axis and the hypothalamic-pituitary-adrenal axis [59]. This endocrine dysregulation is associated with a series of symptoms in AN such as amenorrhea and bone loss. Indeed, AN is usually associated with low bone mineral density and osteoporosis (i.e., skeletal fragility due to bone loss) [60]. In this regard, there are implantable biosensors for monitoring bone health [61]. In other words, biosensors can help monitor a series of biochemicals associated with this endocrine dysregulation, including adipokines and gut peptides related to energy balance, hunger and satiety (e.g., Leptin, Ghrelin, Neuropeptide Y, Peptide YY), hormones related to the menstrual cycle, stress, sleep, and others (e.g., oxytocin, growth hormone, luteinizing hormone, gonadotropin-releasing hormone, progesterone, testosterone, estradiol, cortisol, etc.), and even key processes such as the chronobiology of hormones [2, 62–66]. Clearly, there are many possibilities to integrate implantable biosensors in the healthcare and treatment of AN. However, once again, it is important to evaluate the ethical trade-offs.

Implantable biosensors can also be used in the design of implantable drug delivery systems to release localized and controlled amounts of drugs [2]. Thus, a venue of interest for these biosensors is its use in the design of nanoscale drug delivery systems, such as plant-based nanotechnology (phytonanotechnology) for the delivery of herbal drugs [67, 68]. For example, there is a “renaissance” in the interest for psychedelics like the nonsynthetic ayahuasca, psilocybin, mescaline, peyote [69]. Studies have shown promising effects of psychedelics on key evolved psychological mechanisms like cognitive flexibility [70, 71]. Cognitive flexibility (i.e., the ability to shift perspective to adapt to a changing environment or a new habitat), and in a more general way, behavior flexibility (e.g., to anticipate others' actions and acting accordingly), have evolutive roots that allow developmental adaptation throughout life [72–74]. Individuals with AN display lower cognitive flexibility compared to healthy controls, although most suitable assessment tools are necessary to better explain this deficit and differences [75–77]. Future studies can evaluate the use of biosensors to design implantable drug delivery systems that employ psychedelics such as ayahuasca or psilocybin to enhance key adaptive psychological mechanisms like cognitive flexibility in AN. A similar approach can be used in the design of nutrient delivery systems to improve nutrient bioavailability [78] in individuals with AN.

The article "Sensor Technology and Intelligent Systems in Anorexia Nervosa: Providing Smarter Healthcare Delivery Systems" was published in 2022. Journal: Biomed Res Int.

Other group of implantable biosensors are ingestible sensors for gastrointestinal monitoring [19, 79]. For example, the SmartPill motility testing system (Medtronic) includes a smart pill that travels through the gastrointestinal tract and a software that provides valuable sensor data such as gastric emptying time, colonic transit time, pH, temperature, and pressure from the antrum and duodenum (https://www.medtronic.com/). Other smart pills have been designed to sample the gut microbiome [80]. Individuals with AN present a series of gastrointestinal complications including constipation and bloating, with decreased gastric motility and delayed gastric emptying as the most common underlying causes, although the causes of gastric dysmotility in AN require further research [81]. Regarding the gut microbiota, preliminary results suggest that further research is needed to better characterize the gut microbiome in AN [82–84]. Future research can use ingestible sensors to monitor these gastrointestinal complications and provide a better profile of the gut microbiome in AN.

Finally, an emergent technology of implantable body sensing that is attracting the attention of scientists, inventors, and companies is *smart dust*, considered “the future of humans monitoring” [85]. Based on technologies such as complementary metal-oxide-semiconductor (CMOS) and microelectromechanical systems (MEMS), a smart dust system can consist of thousands of sensor nodes or motes (below 100 *μ*m of size and ultra-low powered), which can sense chemicals, light, magnetism, vibration, acceleration, and temperature [85]. For human monitoring, these sensor nodes can be inserted in the human body (e.g., by drinking water), and neural dust and body dust are probably the most relevant of these technologies for mental healthcare. Neural dust is expected to provide neural recording and neural stimulation [85–87]. However, the present size of these devices (at a millimeter scale) is still a limitation, and brain activity recording via neural dust is still at the conceptual and simulation level [85]. Similarly, body dust is expected to track key biochemical reaction pathways (i.e., metabolic pathways, signaling pathways) involved in human biological systems. Different efforts are being made to downscale the size of these sensors and turn them feasible to produce and use [88, 89]. This advancement in the miniaturization of sensing technologies coupled with nanomaterials with outstanding properties (e.g., graphene composites), optoelectronics (i.e., using light for sensing, recording, stimulating, and controlling), and quantum sensing [9] for the development of optoneuroelectronic or optoelectrophysiology devices [87, 90] could also help bring innovations in this area.

The article "Sensor Technology and Intelligent Systems in Anorexia Nervosa: Providing Smarter Healthcare Delivery Systems" was published in 2022. Journal: Biomed Res Int.

In the future, more individuals with AN could eventually benefit from implantable sensing technology. However, it is important to highlight that the need to use these technologies should be evaluated prior to its implementation in the treatment of AN. In the case they are approved, they should be used under strict regulation to accomplish ethical guidelines and recommendations. Moreover, we suggest that implantable biosensors should not be used as a standalone device, but rather used as the first layer of a smart healthcare system aimed to provide personalized care in the treatment of individuals with AN.

*(2) Epidermal Sensors*. Most biosensors are usually minimally invasive and can monitor, for example, glucose levels [91]. This noninvasive approach is commonly employed to measure physiological signals like pulse or heart rate by attaching sensors to the skin [66]. These epidermal sensors are skin-inspired electronics typically ultrathin, soft, and stretchable, giving the appearance of a second skin or tattoo [10, 66, 92]. An example of this technology is the 5x5mm Lab-on-Skin sensing chip developed by Xsensio (https://xsensio.com), to track biomarkers in human sweat [93, 94]. Similar soft and flexible electrochemical bioelectronics have been developed with the appearance of a wristband or band aid to measure sweat samples [95, 96], wound pH [97], pulse, breath, and body movement [98], among others [10].

Individuals with AN are known to present altered physiological responses to certain stimuli like high-calorie food (e.g., ice cream, pizza) [99] or images of human bodies (e.g., their own body, ultra-thin female bodies) [100]. Therefore, there are several opportunities to use epidermal sensors for the continuous measurement of various physiological responses in AN. For example, electrodermal activity (EDA) sensors to monitor skin conductance response (galvanic skin response), together with epidermal sensors of heart rate, and cortisol, can provide overall a continuous real-time measurement of stress levels, as it can be done with commercial devices [101]. However, it should be noted that epidermal sensors are commercially less developed compared with wearable commercial sensors that have been used more frequently [101, 102]. In any case it is important to highlight that both require a rigorous validation involving the preprocessing of raw data (e.g., noise reduction), signal processing, and feature extraction [103, 104].

*(3) Wearable and Portable Sensors*. Perhaps the most famous sensors among consumers are wearable sensors such as smart watches and portable sensors such as smartphones that incorporate a camera, accelerometer, gyroscope, light detection, etc. The main difference between the epidermal sensors mentioned above and the wearable sensors mentioned here, are that the former are ultrathin, soft, and flexible skin-attached sensors, whereas the latter are commonly rigid and not exclusively used in contact with the skin. Examples of wearable and portable sensor devices include mobile electroencephalography (EEG), smart glasses (including eye-tracker glasses), smart contact lens (rigid, soft), helmet, headband, earring, earpiece, fingertip, rigid wristband, belt, smart textiles (e.g., bra, shirt, sock), and fork [19]. As can be seen, there are different wearable and portable devices, but we will cover just three devices of interest for the healthcare and treatment of AN, prior to covering wearable biosensors.

The article "Sensor Technology and Intelligent Systems in Anorexia Nervosa: Providing Smarter Healthcare Delivery Systems" was published in 2022. Journal: Biomed Res Int.

The first sensor of interest is the portable Sensing Fork designed by Kadomura et al. [105] as part of a mobile based system to promote healthy eating among children. What is interesting about this system is that it integrates several elements of an intelligent system: a sensor, a gamified smartphone application (app), a food type classifier, an eating action classifier, and feedback to the user [105]. A similar device, the HAPIfork, has been developed by the company Hapilabs (https://hapilabs.com).

Mobile EEG sensors are commonly used as a brain-computer interface (BCI) to track brain neural activity [106, 107] and to provide neurofeedback in controlled settings [108, 109] or “in the wild” through mobile phone apps for consumers (e.g., the Muse headband). Although compared to functional magnetic resonance imaging (fMRI), it has a poorer spatial resolution, it has good temporal resolution, it is portable, and inexpensive [110]. The United States has funded research on BCI through “the Defense Advanced Research Projects Agency (DARPA), the Army Research Lab, the Air Force Research Laboratory, and other organizations” [111, 112]. Although most of the funding focused on neuroprosthetics for the treatment of patients with traumatic brain injury, major limb amputation, among others; it had an enormous impact on the development of companies interested in commercializing BCI-based solutions [113]. Among the most popular BCI devices, we have the open hardware OpenBCI, the Emotiv EPOC, the Muse headband, and the NeuroSky's EEG biosensor.

Eye-trackers are other well-known sensors used for various purposes including research on advertising [114, 115], gender attitudes [116], body-related attentional bias [117], and eating disorders [118–121]. Although desktop eye-tracking devices are by far more precise, wearable eye-trackers provide descent resolution and sampling rates [122]. Popular eye-trackers include Pupil Labs glasses, Tobii glasses, SMI glasses, and low-cost solutions like RemoteEye [123].

Finally, wearable biosensors employ a biological recognition element (receptor) and a transducer (e.g., electrode) to detect biofluids [124, 125]. Biosensors can use different receptors, such as enzymatic electrochemical biosensors to detect glucose, uric acid, lactate, and hydrogen peroxide; intact living cells to work as cell sensors and microbial sensors; antibodies to act as immunosensors; and even nucleic acids (e.g., aptamers) to recognize molecules [125]. Therefore, wearable biosensors can have different functionality, such as detecting metabolic parameters (e.g., pH, electrolytes), physiological signals (e.g., heart rate, skin temperature), and even toxic chemicals like organophosphate compounds [126]. A recent review of electrochemical affinity biosensors details a series of devices to detect hormones and metabolites that can be of relevance for the treatment of AN, like the aforementioned cortisol, leptin, ghrelin, growth hormone, estradiol, among others [65].

Wearable biosensor devices worth mentioning include contact lenses and eyeglasses for tear biosensing [127, 128], the 61 x 41 x 5.5 mm VivaLINK (https://www.vivalink.com/) axillary patch to measure temperature, the 90 x 20 x 7.9 mm cardiac patch from the same company, textile sensors (smart textile) for sweat analysis [129], to name just a few. In fact, the list of wearable biosensors and their applications is so extensive that we refer the reader to previous work [19, 66, 103, 124, 126, 130–133].

#### 1.1.2. Sociometric Sensors

The quantity and quality of interpersonal relationships exert a strong influence in shaping the individual's affect, cognition, and behavior. Social network analysis has been used for a long time to study human social interaction [134]. Traditional sociometric techniques employ self-reports about friendships and networks, providing a valuable but limited view of human interactions [135]. In this regard, computational science methods that include sensing technology, social physics, and simulations can provide accurate measures of human social interaction and remarkably precise predictions of individual and collective human behavior [136, 137]. Therefore, in this group, we consider as a sociometric sensor any sensor (i.e., implantable, epidermal, wearable, portable) that can provide relevant social data.

The article "Sensor Technology and Intelligent Systems in Anorexia Nervosa: Providing Smarter Healthcare Delivery Systems" was published in 2022. Journal: Biomed Res Int.

For example, the growing adoption of 5G technology and pervasive wireless sensors in smart spaces (i.e., smart cities, smart organizations including smart hospitals, and smart homes) provide a fine-grained collection of social signals, allowing a continuous remote monitoring of human daily life activities and social interactions. In this scenario, sociometric sensor devices have been developed to provide accurate measures of interpersonal proximity and verbal communication [138–141^]^. Sociometric data collected by sensors in daily life settings can be used to examine peer processes and family processes in AN with the possibility to identify cliques (e.g., group of friends), influence agents in the network, and key communication and interaction processes known to shape social norms within groups [142]. Similarly, sociometric sensors can be used to examine group interactions, communication, collaboration, and overall group dynamics [143] among healthcare professionals [144]. In sum, methodologies from computer science and social sciences (i.e., computational social sciences) can be employed for social data mining (e.g., using sociometric sensors), social signal processing [145], simulation (e.g., agent-based models), and interventions [146].

#### 1.1.3. Ambient Sensors

In this category, we basically have outdoor and indoor ambient sensors. Regarding outdoor sensors, many urban cities are equipped with environment-embedded sensors to measure physical conditions such as humidity, temperature, atmospheric pressure, and wind for weather forecasting. In fact, there are several types of outdoor sensors: soil moisture sensors for irrigation management; air quality sensors to track pollution; and city cameras, including thermal cameras and AI cameras, for security, traffic management, people counting, monitoring energy transformers to avoid overheating, etc.

Along with these sensors, we have satellite data, location data, and a geographic information system (GIS) to, for example, map the surrounding built environment of citizens. Although all these data from ambient sensors and geolocation apparently seem disparate, we can use computer vision, signal processing, simulation, machine learning and AI, to analyze a built environment, identify patterns like individual and group human behavior within cities, and predict future patterns [147].

The article "Sensor Technology and Intelligent Systems in Anorexia Nervosa: Providing Smarter Healthcare Delivery Systems" was published in 2022. Journal: Biomed Res Int.

The built environment of a neighborhood has an important effect on health behaviors. For example, built environments can facilitate open air physical activity if they provide suitable infrastructure like walking paths [148]. Similarly, healthy food availability and accessibility in living surroundings can facilitate healthy eating [149]. Individuals with AN struggle with food and it could be even worse if the surrounding living environment does not provide healthy food choices (e.g., the so-called “food deserts”) or food that fits a personally tailored nutrition [150, 151]. Furthermore, high levels of physical activity are common in individuals with AN [152, 153], and this overactivity has been linked to thermoregulation and ambient temperature [154], both of which can be measured with sensors.

Therefore, environment-embedded sensors can be implemented in indoor and outdoor spaces to measure diverse conditions like temperature, ambient radio signals (e.g., Wi-Fi), air quality, location, etc. Then, we can integrate the information of the built environment that surrounds individuals with AN with the data of their indoor living conditions, into intelligent systems for healthcare monitoring. For example, weather forecasting data with previous individual's mobility and sleep patterns [155] could predict physical overactivity in outdoors in AN. An intelligent system that integrates this information together with real-time air quality data [156] can send an SMS reminder to the user to avoid excessive exercise and reduce his exposure to air pollution, the latter linked to cardiovascular diseases [157, 158]. In a similar fashion, data from global positioning system (GPS) and ecological momentary assessment (EMA) has been used to monitor the food environment and food and eating patterns [159].

As we will see below [160], there are many other opportunities to integrate ambient sensors in intelligent systems for healthcare monitoring.

### 1.2. Intelligent Systems

Intelligent systems for healthcare monitoring can be designed to relieve the burden of healthcare professionals, reduce costs, and improve the treatment of individuals with AN. In this regard, it is important to integrate sensor data with traditional data from the clinical history and physical examination, laboratory tests, self-reports, etc. For example, Figure 1 shows an intelligent system that employs machine learning models integrating sensor data and traditional data (e.g., self-reports) to provide feedback to the caregiver, physician, and patient.

The article "Sensor Technology and Intelligent Systems in Anorexia Nervosa: Providing Smarter Healthcare Delivery Systems" was published in 2022. Journal: Biomed Res Int.

First, given that we can acquire data from multiple sensors, sensor fusion is recommended to enhance the quality of the data collected by the sensors [161]. For example, if the signal of a heart sensor is affected by noise (e.g., movement), heart data from additional sensors can ensure the reliability of heart monitoring [161]. Similarly, sensor fusion can be used to obtain data that cannot be obtained by isolated sensor data [161].

Then, the architecture to process these multisensor sensor data can be a decentralized distributed architecture [162, 163], like a network of nodes with a hierarchical structure. For example, we can employ Wireless Sensor Networks (WSNs), which are networks of scattered wireless sensors to collect diverse physical data from the environment [164], together with Wireless Body Area Networks (WBANs) that comprise body sensors located in different parts of the body [98, 161]. The first layer in this hierarchy constitutes the edge computing layer that retrieves the data from body sensors, RFIDs, etc. These data are forwarded to a fog computing layer (e.g., a Raspberry Pi, a smartphone), which acts as the connecting link between the edge layer and the cloud computing (the highest layer in this hierarchy), reducing latency and enhancing efficiency [165]. Finally, cloud computing can be leveraged to perform the most arduous tasks, including the use of artificial intelligence (e.g., graph neural networks) for classification and predictive analytics.

Although, the need to use cloud services should be evaluated in terms of cybersecurity, privacy, confidentiality, and environmental sustainability [162]. Moreover, improvements in radio technology (e.g., 6G standard, autonomous, dynamic, distributed, adaptive wireless networks), will allow more efficient infrastructures depending less on remote cloud services. For example, Amazon Web Service (AWS) Wavelength (https://aws.amazon.com/wavelength/features/) is a mobile edge computing infrastructure that embeds AWS services within 5G networks, reducing the need for mobile applications to heavily rely on remote cloud servers.

There are several examples of a three-layer architecture for healthcare monitoring. Niu et al. [98] developed the bodyNET system that employs five wearable epidermal sensor nodes and smart textiles that operate with a smartphone via Bluetooth, and a cloud server via cellular network, for pulse detection, breath detection, and body movement detection. Similar systems have been used for tracking eating behavior [166] to predict heart failure [167, 168] and mental health issues such as depression [169].

The article "Sensor Technology and Intelligent Systems in Anorexia Nervosa: Providing Smarter Healthcare Delivery Systems" was published in 2022. Journal: Biomed Res Int.

However, perhaps the most promising venue of intelligent systems in healthcare is to provide tailored interventions at real-time using mobile health (mHealth) technology, digital twin (e.g., a digital replica of a patient), social robotics, or others. That is the case of digital just-in-time adaptive interventions (JITAIs) or ecological momentary interventions [170–174] that can adopt a *human-aware* AI (or human-centered AI, i.e., AI systems that are centered on the user) approach [175] and a *context-aware* approach [168, 174]. In this case, these intelligent systems are grounded in both evidence-based interventions (e.g., behavior change theories) and continuous learning (e.g., reinforcement learning), to provide a user-friendly experience tailored to the needs of the user. For example, a JITAIs can be a gamified mobile app grounded in Cognitive Behavioral Therapy (CBT), and the mechanisms of behavior change [176, 177] that delivers reminders or instructions to support decision making, behavior change, activities of daily life, etc. These alerts can benefit individuals with AN and those monitoring their treatment [170]. Sensing technologies can be key in designing these intelligent systems, and these systems can be integrated together with traditional interventions to provide a smarter healthcare in AN.

## 2. Discussion

This review focused on the integration of sensor technology and intelligent systems, to provide smarter healthcare delivery systems in Anorexia Nervosa (AN). Through this narrative review, we have seen that to design and deploy these intelligent systems, we require the effort of professionals from diverse fields. Domain expertise in the field of eating disorders, healthcare management, sensor technologies, internet of things (IoT), big data, data science, artificial intelligence is required, among others. However, global challenges such as the COVID-19 pandemic or climate change, have demonstrated that the deployment of intelligent systems is feasible through cooperation and consilience across different disciplines, and it fosters innovation scaling [178].

Current interventions that use technology, particularly mobile technology (i.e., mHealth interventions) for the treatment of eating disorders such as AN are scarce, but the use of evidence-based techniques, gamification, and the possibility of remote monitoring and guidance are just some of the factors that can make them attractive for patients and clinicians [179–182]. Therefore, as we have seen previously, there are several opportunities to integrate sensing technology and foster innovation in the field of eating disorders, particularly in healthcare settings. Anorexia Nervosa affects the lives of millions of women and is a chronic condition that deserves the careful attention of health professionals but can create a burden among them. Sensing technologies can relieve this burden if they are used to not only provide data but also used particularly if they are embedded in intelligent systems for smarter healthcare of patients with eating disorders.

The article "Sensor Technology and Intelligent Systems in Anorexia Nervosa: Providing Smarter Healthcare Delivery Systems" was published in 2022. Journal: Biomed Res Int.

In this regard, we highlight the fact that there is a fast development in the manufacture of new and low-cost electronic devices, particularly in modern cities like Shenzhen (China). We have mentioned above that these new technologies, like polymer and graphene composite-based nanosensors, quantum sensors, will be the future of human monitoring. As we also mentioned, there are ethical concerns that arise from ubiquitous technologies. However, we must also mention environmental and sustainability issues related to the manufacture of sensor technologies. For example, intelligent cameras with computer vision capabilities can be used for healthcare but require higher power consumption and materials like lithium or gold, that usually have high and hidden environmental costs. In summary, it is important to recognize along the ethical issues mentioned above, the environmental sustainability of the manufacture and use of these sensors. Future research should consider alternatives to man-made sensors, such as nature-based biosensors. For example, plants used as sensors (phytosensors), are a more sustainable alternative, have higher sensitivity and specificity, and can be used for human monitoring [183, 184].

Finally, we have shown how sensor technologies can be integrated in the treatment of AN through the design and deployment of intelligent systems supported by artificial intelligence. In this regard, it is worth mentioning that there are established network standards (e.g., IEEE 802.15.6 for WBANs), device standards (e.g., IEEE/ISO 11073-10420-2010 for body composition analysis), and communication standards (e.g., Proxy Mobile IPv6, PMIPv6 by the Internet Engineering Task Force, IETF) for these systems. However, to implement more advanced and future intelligent systems, we need to design new standards and protocols that require the collaboration and synergy of different professionals. To give an example, there is a joint effort to build cyberphysical social systems, which includes what is called Societies 5.0, a new paradigm to modeling and managing complex systems such as societies [185, 186]. The transition towards these cyberphysical social systems, and more particularly cyberphysical medical systems [187], urgently requires interdisciplinary collaboration [188]. For example, there are cybersecurity issues, like cyberattacks to healthcare devices [187], that can be solved with secured protocols and standards [189, 190]. Importantly, cyberphysical social systems can be used for behavior monitoring [191], and therefore they have a great potential for smarter healthcare at the individual and population level.

The article "Sensor Technology and Intelligent Systems in Anorexia Nervosa: Providing Smarter Healthcare Delivery Systems" was published in 2022. Journal: Biomed Res Int.

## 3. Conclusions

In conclusion, sensing technologies and intelligent systems can be designed and deployed for smarter healthcare for AN. However, there are technical, ethical, and environmental sustainability issues that must be considered prior to implementing these systems. A joint collaboration of professionals and other members of the society involved in the healthcare of individuals with AN can help in the development of these systems. The evolution of cyberphysical systems should be considered in these collaborations.

## Figures and Tables

**Figure 1:** An intelligent integrated system for healthcare monitoring. Note: EHR=Electronic health records. Image icons are from The Noun Project, 2022. (https://thenounproject.com/). Royalty-free license.
